# Immobilization of metribuzin-degrading bacteria on biochar: Enhanced soil remediation and bacterial community restoration

This article has been retracted.

**DOI:** 10.3389/fmicb.2022.1027284

**Published:** 2023-02-15

**Authors:** Abdul Qadeer Wahla, Samina Anwar, Muhammad Irfan Fareed, Wasiq Ikram, Liaqat Ali, Hesham F. Alharby, Atif A. Bamagoos, Afaf A. Almaghamsi, Samina Iqbal, Shafaqat Ali

**Affiliations:** ^1^Soil and Environmental Biotechnology Division, National Institute for Biotechnology and Genetic Engineering College, Pakistan Institute of Engineering and Applied Sciences (NIBGE-C, PIEAS), Faisalabad, Punjab, Pakistan; ^2^Department of Life Sciences, School of Science, University of Management and Technology, Johar Town, Lahore, Pakistan; ^3^School of Botany, Minhaj University Lahore (MUL), Lahore, Pakistan; ^4^Department of Biology, University of Okara, Renala Khurd, Okara, Pakistan; ^5^Department of Soil and Environmental Sciences, University of Agriculture Faisalabad, Sub Campus Burewala, Vehari, Pakistan; ^6^Department of Biological Sciences, Faculty of Science, King Abdulaziz University, Jeddah, Saudi Arabia; ^7^Plant Biology Research Group, Department of Biological Sciences, Faculty of Science, King Abdulaziz University, Jeddah, Saudi Arabia; ^8^Department of Biology, College of Science, University of Jeddah, Jeddah, Saudi Arabia; ^9^Department of Environmental Science, Government College University, Faisalabad, Pakistan; ^10^Department of Biological Sciences and Technology, China Medical University, Taichung, Taiwan

**Keywords:** Bioaugmentation, Rice-husk biochars, Biodegradation, Metagenomics analysis, Soil Bacterial diversity

## Abstract

Metribuzin (MB), a triazinone herbicide is extensively sprayed for weed control in agriculture, has been reported to contaminate soil, groundwater, and surface waters. In soil, MB residues can negatively affect not only the germination of subsequent crops but also disturb soil bacterial community. The present study describes the use of biochar as a carrier material to immobilize MB-degrading bacterial consortium, for remediation of MB-contaminated soil and restoration of soil bacterial community in soil microcosms. The bacterial consortium (MB3R) comprised four bacterial strains, i.e., *Rhodococcus rhodochrous* AQ1, *Bacillus tequilensis* AQ2, *Bacillus aryabhattai* AQ3, and *Bacillus safensis* AQ4. Significantly higher MB remediation was observed in soil augmented with bacterial consortium immobilized on biochar compared to the soil augmented with un-immobilized bacterial consortium. Immobilization of MB3R on biochar resulted in higher MB degradation rate (0.017 Kd^−1^) and reduced half-life (40 days) compared to 0.010 Kd^−1^ degradation rate and 68 day half-life in treatments where un-immobilized bacterial consortium was employed. It is worth mentioning that the MB degradation products metribuzin-desamino (DA), metribuzin-diketo (DK), and metribuzin desamino-diketo (DADK) were detected in the treatments where MB3R was inoculated either alone or in combination with biochar. MB contamination significantly altered the composition of soil bacteria. However, soil bacterial community was conserved in response to augmentation with MB3R immobilized on biochar. Immobilization of the bacterial consortium MB3R on biochar can potentially be exploited for remediation of MB-contaminated soil and protecting its microbiota.

**Graphical Abstract:** 

## Introduction

Metribuzin (abbreviation MB; CAS number 21087-64-9) is a triazinone herbicide that is applied in agriculture to obstruct the growth of weeds *via* disrupting photosystem II (Zhang et al., 2014). Due to weak sorption to soil particles and high water solubility (1.05 g L^−1^), MB has the potential to contaminate run-off water and seep into to groundwater, and thus pollute surface as well as subsurface water bodies (Honorio et al., 2013). It is well established that metribuzin and its metabolites are a significant hazard to natural aquatic systems as well as non-targeted algae and macrophytes (Ara et al., 2013; Kumar et al., 2017). In soil, MB residues negatively affect the development of some rotating crops, and on the structure of soil microbes and other life forms (Bedmar et al., 2004; Kucharski et al., 2016; Huang et al., 2018). The negative effect of MB on the abundance and activity of soil microorganisms has been documented by Latha and Gopal, 2010; (Mehdizadeh et al., 2019; Yang X. et al., 2019; Cara et al., 2021).

The global concern about the existence of MB residues in soil and water has prompted researchers for exploration of approaches for alleviation of this pesticide from cultivated soils. Bioremediation is a promising strategy that exploits the capability of microorganisms to remediate pollutants from contaminated matrices in an effective, non-hazardous, cheap, easily adaptable, and environment friendly (Verma et al., 2014; Tarfeen et al., 2022).

Largely, the efficiency of bioremediation depends on the degradation capacity of indigenous or exogenous microbes and favorable environmental conditions for their growth and activity (Anwar et al., 2022). Yet, given the aforementioned negative impact of MB on soil microbial communities, it is conceivable that high *in situ* MB concentrations hamper its degradation kinetics (Kaur et al., 2022). Furthermore, MB-transformation capabilities of autochthonous soil microbial communities appear to be generally low (Magan et al., 2022).

Bioremediation through bioaugmentation of exogenous contaminant-degrading microbes to the polluted soil may improve pesticide degradation. However, this method has several drawbacks, including limited microbial survival, proliferation, mechanical disturbances, limited nutrient availability, low adaptability, and competition with indigenous microorganisms (Boopathy, 2000). An alternate strategy is to encapsulate exogenous contaminant-degrading bacteria on a carrier material, which can serve as an optimal site for their survival and functioning under biotic (competition, predation) and abiotic soil conditions (Chen B. et al., 2012; Huang et al., 2015). An excellent immobilization carrier not only provides a suitable environment for microbial colonization but also plays an essential role in enhanced pollutant sorption, and degradation thereafter (Lu et al., 2018).

The present study hypothesized that biochar would act as an ideal carrier for metribuzin-degrading bacteria, to enhance the removal of metribuzin from soil as compared to freely applied bacteria. Biochar has already been considered a promising carrier material to immobilize bacteria for enhanced remediation efficiency of the contaminated soils (Liu et al., 2017; Yang Y. et al., 2019). Use of biochar as soil additive to improve soil health and soil fertility, to sequester carbon, and enhance agricultural production is also well established (Atkinson et al., 2010; Wang et al., 2016).

The objective of the present research was to evaluate the bioremediation potential of MB-degrading bacterial consortium MB3R immobilized on biochar in soil microcosms. This work highlights the negative effect of metribuzin on the soil microbial community, and demonstrates that these effects can be reversed by augmentation of the soil with the biochar-immobilized bacterial consortium MB3R. The novelty of the work is depicted by the fact that there is no single report available about the application of bacterial consortium immobilized on biochar for the removal of MB from soil with the simultaneous investigation of changes in soil microbial community structure.

## Materials and methods

### Chemicals

Metribuzin (technical grade, 97.6% purity) was obtained from Tara Crop Sciences (Lahore, Pakistan). Analytical grade MB (99.9% purity), metribuzin-desamino (abbreviation DA; CAS number 35045-02-4), metribuzin-diketo (DK; CAS number 56507-37-0) and metribuzin-desamino-diketo (DADK; CAS number 52236–30-3) were acquired from Dr. Ehrenstorfer GmbH (Germany). All other chemicals including acetonitrile, methanol, and methylene dichloride (DCM; all of HPLC grade) were procured from Sigma Aldrich (Germany).

### Metribuzin-degrading bacterial consortium MB3R

The MB-degrading bacterial consortium MB3R comprising *Rhodococcus rhodochrous* strain AQ1, *Bacillus tequilensis* strain AQ2, *Bacillus aryabhattai* strain AQ3, and *Bacillus safensis* strain AQ4 was established in our lab earlier as reported previously (Wahla et al., 2019). The strains were stored individually in 15% (v/v) glycerol stocks at −80°C, and revived when required. Before the formation of bacterial consortium MB3R, the compatibility of all bacterial strains was checked by cross streak method (Santiago et al., 2017). All strains were found compatible with each other. Strains were cultured in Lysogeny Broth (LB) individually at 30°C overnight, harvested by centrifugation at 5000 × g and 4°C for 10 min, and suspended in autoclaved normal saline solution (0.85% w/v) to an optical density at 590 nm wavelength (OD_590_) of 1.00 with the following cell densities: strain AQ1 with 7 × 10^7^ Colony-Forming Units, CFU mL^−1^, strain AQ2 with 5 × 10^7^ CFU mL^−1^, strain AQ3 with 5 × 10^7^ CFU mL^−1^, and strain AQ4 with 4 × 10^7^ CFU mL^−1^. These suspensions were mixed to generate 7 × 10^7^ CFU ml^−1^ of MB3R.

### MB3R-biochar formulation

Biochar was made from rice husk *via* pyrolysis (Khorram et al., 2016) at the Soil Fertility Laboratory, Institute of Soil and Environmental Sciences, University of Agriculture Faisalabad, Pakistan. The consortium MB3R was adsorbed on biochar as described earlier (Liu et al., 2017). Briefly, the biochar and MB3R cell suspension was mixed at a 5:100 (w/v) ratio and incubated at 30°C with shaking at 150 rpm on a rotary shaker for 24 h. The rate of bacterial consortium onto biochar was determined in triplicate *via* comparing the OD_590_ reduction of MB3R suspensions in the presence of biochar vs. the reduction in normal saline solution. For the former, suspensions were centrifuged at 5000 × g for 10 min and the OD_590_ of the supernatant was determined. The adsorption effectiveness was calculated by the following formula (Li et al., 2017).


(1) $$\begin{array}{l} \%\;\mathrm{Adsorption of}\;\\ \mathrm{MB}3R\;\mathrm{on}\;\mathrm{biochar}=\left({\mathrm{OD}}_{\mathrm{BC}}\times {\mathrm{OD}}_{\mathrm{NS}}\right)/{\mathrm{OD}}_{i}{}^{2}\times 100 \end{array}$$

OD_BC_ = OD_590_ of the MB3R-biochar supernatant after 24 h

OD_NS_ = OD_590_ of the MB3R suspension in normal saline after 24 h

OD_i_ = initial OD_590_ of bacterial suspension;

The efficacy of MB3R adsorption on biochar was analyzed as 50%. The MB3R-biochar formulation pellets were stored at 4°C until further use in soil inoculation studies.

### Collection and spiking of soil with metribuzin

Soil free of metribuzin residues was collected from a field located at wheat research fields, Ayub Agricultural Research Institute (AARI), Faisalabad (31.4504° N, 73.1350° E), Pakistan. After air drying and sieving, the soil was studied for standard physical and chemical properties (Table 1). MB (technical grade) was applied to the soil by adopting a method reported previously (Brinch et al., 2002) with little modifications. Briefly, the MB solution (1% in acetonitrile) was mixed thoroughly with sand in a small desiccator. The evacuation pressure in the desiccator was kept 50 mbar until the solvent was evaporated. The spiked sand was mixed prudently into the collected soil to achieve the final MB concentration 2.5 mg kg^−1^ soil.

**Table 1:** Physio-chemical properties of soil used in MB biodegradation microcosm studies.

Sr. no.	Treatments	Remarks
1	pH	8.3
2	Electrical conductivity (EC, dS m^−1^)	6.2
3	Total nitrogen (%)	0.052
4	Phosphorus (ppm)	6.9 ppm
5	Potassium (ppm)	120 ppm
6	Organic matter (%)	1.05%
7	Sand (%)	29
8	Silt (%)	47.5
9	Clay (%)	23.5
10	Texture class	Clay loam

### Experimental layout

Microcosm experiments were carried out to assess the potential of MB3R to degrade MB in soil when applied as suspensions and as biochar formulation. Two independent rounds of experiments with individual soil samples (termed 1st and 2nd experiment) with three replicates per microcosm were conducted to ensure the reproducibility of results. The experiments comprised four treatments at initial metribuzin concentration of 2.5 mg kg^−1^ soil. The experiments were conducted in plastic boxes (2.5 cm width × 2.5 cm length is × 21 cm height) containing 2.0 kg soil using a completely randomized design. Experiments consisted of the following treatments.

1. unamended soil (labeled “Control”).

2. MB-contaminated soil (labeled “S-UI”).

3. MB-contaminated soil augmented with biochar (labeled “S-UI-BC”).

4. MB-contaminated soil augmented with 1 × 10^5^ CFU MB3R g^−1^ soil (labeled “S-I”).

5. MB-contaminated soil augmented with 2 g MB3R-biochar kg^−1^ (labeled “S-I_BC”).

For the determination of residual MB and its metabolites (see Section 2.3.1), soil samples were taken 30, 60, and 90 days after inoculation (DAI). To evaluate the effect of MB and MB3R adsorbed onto biochar on the soil bacterial community, soil samples (*n* = 3) were collected at the end of the 2nd experiment using a sterile spatula and stored at −80°C until further processing.

### MB and its metabolites in soil

MB and its metabolites DA, DK, and DADK were extracted from soil samples as described earlier (Anwar et al., 2009). Briefly, soil samples (10 g) were extracted with equal volume of methylene dichloride twice, aspirated under nitrogen, dissolved in acetonitrile (1 ml), and filtered through a 0.45 μm filter before analysis by HPLC. A Dionex UHPLC system (Thermo Scientific, Sunnyvale, CA, United States) equipped with a DAD 3000 RS detector, LPG 3000 quaternary pump, WSP 3000 TRS autosampler, degasser, and column oven was used. Chromeleon 7.0 software was used for data recording and processing. The chromatographic separation was performed using a reverse-phase ODS2 C18 column (Thermo Hypersil gold^™^, 250 × 4.6 mm). Separation was achieved using the mobile phase consisting of acetonitrile: water (45:55) acidified with acetic acid (0.5%) with a flow rate of 0.4 ml min^−1^. The injection volume was 15 μl, and deionized water was used as the injection washing solution. The detector wavelength was set at 280 nm for the determination of MB and its metabolites. The retention time of the MB, DA, DK, and DADK was 6.9, 5.2, 4.3, and 4.5 min, respectively. Standard curves were drawn by plotting peak areas versus concentrations of MB, DA, DK, and DADK analytical standards dissolved in acetonitrile at 1.25, 2.5, 5.0, 7.5, 10, 20, 40, and 50 mg L^−1^.

### MB degradation kinetics and statistical analysis

Kinetic analysis for MB biodegradation in soil was carried out by plotting ln [C_t_/C_0_] against time of incubation. MB degradation rate constant (k, h^−1^) and half-life (T_1/2_, days) were determined using the following equations.


(1) $$C_{t}=C_{0}\times e{-}^{\mathrm{kt}}$$

(2) $$T_{1/2}=\ln\;\left(2\right)/k$$

C_t_ and C_0_ denote concentrations of MB (mg L^−1^) at time “t” and time “zero” respectively.

Minitab 17 software was used for the statistical analysis of data related to MB residues and bacterial population in soil. Further, the significance of results (*p* < 0.05) was confirmed by employing Tukey’s test.

### Nucleic acid-based analysis of the soil bacterial community

The structure of the bacterial community in soil samples was analyzed *via* Illumina-based amplicon sequencing of the bacterial 16S rRNA gene. First, the Power Soil DNA Isolation Kit (MP BIO Laboratories) was used to extract total soil DNA by following the manufacturer instructions. The quality and quantity of DNA were checked by agarose gel (2%) and Qubit fluorometer (Invitrogen) respectively. Next, the 16S rRNA gene (V1-V2 hypervariable region) was amplified by PCR using the 27F (5’ AGAGTTTGATCCTGGCTCAG 3′) and 338R (ATGCTGCCTCCCGTAGGAGT) primers (Etchebehere and Tiedje, 2005; Yu et al., 2013). The amplicons were pooled and used to generate Illumina pair-end libraries by targeting the hypervariable region V1-V2 of the 16S rRNA and paired-end sequenced (2 × 250 bp) on an Illumina MiSeq platform (San Diego, California, United States). Image analysis and base calling were accomplished using the Illumina Pipeline. Then, raw reads were merged by the Ribosomal Database Project (RDP) assembler, and the MOTHUR pipeline (based on SILVA reference database, Gotoh algorithm) was used for the alignment of sequences (Schloss et al., 2009; Quast et al., 2012; Cole et al., 2013). All reads were trimmed to remove primer and barcode nucleotide sequences. Before further analysis, pre-clustering and filtration (sequence length ≥ 250 bp and the average abundance of ≥0.02%) of sequences were carried out using Mothur to produce phylotypes. The phylotypes were analyzed by naïve Bayesian RDP classifier (pseudo-bootstrap threshold of 80%) to assign taxonomic ranks (Wang et al., 2007). The shiny-ampvis2 package was used for the determination of relative abundance, alpha and beta diversity of phylotypes based on whole OTU composition (Andersen et al., 2018).^1^ The alpha diversity indices Chao1, Shannon, and Simpson were determined for comparing the richness, evenness, and diversity of the various treatments. Principal component analysis (PCA) was used to compare the values of beta diversity of soil bacterial community, and Microsoft Excel 2016 was used for making bar plots, respectively.

## Results

### Biodegradation of metribuzin by the consortium MB3R

As deduced from residual MB concentration in soil, MB degradation was 24.30 and 25.96% in soil inoculated with MB3R (S-I) as compared to uninoculated soil (S-UI) where only 9.60 and 7.20% of MB degradation was observed after 30 days during 1st and 2nd experiment, respectively (Figure 1). The augmentation of spiked soil with MB3R immobilized on biochar (S-I_BC) further enhanced MB degradation as 42.07 and 40.92% degradation were observed in 1st and 2nd experiments, respectively, after 30 days (Figure 1).

**Figure 1:** Biodegradation of metribuzin (MB) soil under various treatments at 30, 60 and 90 days after incubation (DAI) during two experiments. Initial MB concentration in the soil was 2.5 mg Kg^−1^ and % degradation was calculated based on residual concentration.

After the end of each experiment, 78.37 and 75.09% MB removal was observed in treatment S-I_BC in contrast to treatment S-I where 59.90 and 61.73% degradation occurred (Figure 1). In treatment S-UI, the MB removal was only 24 and 26% at the end of both experiments (after 90 days of incubation). The results demonstrated that the immobilization of the bacterial consortium MB3R on biochar played a significant role for remediation of soils contaminated with MB.

### MB degradation kinetics

In soil, MB degradation during both experiments followed first-order kinetics. The MB degradation rate constant (Kd^−1^) in soil spiked with 2.5 mg L^−1^ MB (S-UI) during both experiments was only 0.003. Addition of biochar alone (S-UI-BC) slightly increased MB degradation (Kd^−1^ = 0.004–0.005). However, MB3R inoculation significantly increased MB degradation rate (*p* < 0.05). In treatments S-I and S-I_BC, the MB degradation rate constants were 0.010 and 0.017, respectively, during both experiments (Table 2).

**Table 2:** Metribuzin (MB) degradation kinetics in soil under various treatments.

Treatments	Regression equation		Rate constant (Kd^−1^)		Half-life (T_1/2_, days)		Regression coefficient (R_2_)	
	1st Exp	2nd Exp	1st Exp	2nd Exp	1st Exp	2nd Exp	1st Exp	2nd Exp
S-UI	C_t_ = 2.5e^-0.003^	C_t_ = 2.5e^-0.003^	0.003	0.003	218.9	204.3	0.9988	0.9911
S-UI**_**BC	C_t_ = 2.5e^-0.005^	C_t_ = 2.5e^-0.004^	0.005	0.004	152.4	168.4	0.9931	0.9655
S-I	C_t_ = 2.5e^-0.010^	C_t_ = 2.5e^-0.011^	0.010	0.011	68.1	64.9	0.9909	0.9967
S-I**_**BC	C_t_ = 2.5e^-0.017^	C_t_ = 2.5e^-0.015^	0.017	0.015	40.7	44.7	0.9987	0.9972

S-UI = Metribuzin-contaminated soil.

S-UI_BC = Metribuzin-contaminated soil supplemented with biochar.

S-I = Metribuzin-contaminated soil inoculated with bacterial consortium MB3R.

S-I_BC = Metribuzin-contaminated soil inoculated with bacterial consortium MB3R immobilized on biochar.

The half-life (T_1/2_) of MB in untreated soil (S-UI) was 218 and 204 days during the 1st and 2nd experiment, highlighting its persistence in soil (Table 2). The treatment of soil with the MB-degrading bacterial consortium MB3R (S-I) reduced the half-life to 68 and 64 days, which was further reduced to 44 and 40 days in treatments where the bacterial consortium immobilized on biochar (S-I_BC) was applied (Table 2). These results demonstrated that the augmentation with the MB3R consortium-biochar formulation can be used as a practical approach for the restoration of MB-contaminated soils.

### Detection of MB metabolites

Three metabolites of metribuzin, desamino-metribuzin (DA), diketo-metribuzin (DK), and desamino-diketo-metribuzin (DADK) were detected only in MB-contaminated soil treated with the consortium MB3R alone (S-I) and MB3R immobilized on biochar (S-I_BC). Maximum residual concentrations of DA, DK, and DADK were found in soil at 30 days after incubation (DAI) and lowest at 90 DAI (Figure 2). The concentration of MB in treatment S-I_BC was lower, while concentrations of DA, DK, and DADK were higher as compared to treatment S-I in all samplings. A gradual decrease in the amounts of MB, DA, DK, and DADK was observed at 60 and 90 DAI than 30 DAI, which indicates that the bacterial consortium MB3R also has potential to degrade MB metabolites.

**Figure 2:** Residual concentrations (mg Kg^−1^) of metribuzin (MB) and its metabolites i.e., desamino-metribuzin (DA), diketo-metribuzin (DK) and desamino-diketo-metribuzin (DADK) in soil under various treatments at 30, 60 and 90 days after incubation (DAI).

### Effect of MB and biochar additions on soil microbial community

The effect of MB, biochar, and the bacterial consortium MB3R (alone and in combination with biochar) on soil bacterial communities was assessed by the analysis of 16S rRNA gene amplicon sequences. The diversity of the soil bacterial community under various treatments was analyzed by calculating the alpha diversity indices Chao1, Shannon, Simpson, and Fisher (Table 3). The bacterial alpha diversity indices Shannon, Simpson, and Fisher indicated that alpha diversity was not significantly different (*p* < 0.05) between the treatments. In contrast, beta diversity analysis of OTU profiles using principal component analysis PCA showed that treatments S-UI and S-I were different from the control (C), S-UI_BC, and S-I_BC treatments (Figure 3). The sample clustering was based on ~78.2% of the data variance by the first two principal components (factors), i.e., 46.7 and 31.5%, respectively. These results indicate that the addition of biochar provided a stabilizing effect on the bacterial community when challenged with MB.

**Table 3:** Alpha diversity metrics of soil bacterial communities in different treatments.

Treatments	Observed	Chao1	Shannon	Simpson	Fisher
C	1671b (45)	1751b (49)	6.76a (0.72)	0.998a (0.07)	392a (17.32)
S-UI	1672b (30)	1746b (37)	6.17a (0.48)	0.990a (0.05)	366a (08.66)
S-UI_BC	1898a (39)	2123a (69)	6.43a (0.51)	0.991a (0.06)	438a (24.25)
S-I	1736ab (52)	1818b (58)	6.40a (0.56)	0.994a (0.08)	371a (14.43)
S-I_BC	1741ab (43)	1826b (42)	6.44a (0.38)	0.993a (0.05)	364a (19.05)

C = Native soil.

S-UI = Metribuzin-contaminated soil.

S-UI_BC = Metribuzin-contaminated soil supplemented with biochar.

S-I = Metribuzin-contaminated soil inoculated with bacterial consortium MB3R.

S-I_BC = Metribuzin-contaminated soil inoculated by immobilized bacterial consortium MB3R with biochar as carrier.

Each value is mean of three replicates; standard error of the replicates is presented in parenthesis (±). Means followed by different letters are significantly different (p < 0.05).

**Figure 3:** Beta-diversity analysis of soil microbial communities under various treatments by using principal component analysis (PCA) based on Operational Taxonomic Units (OTUs).

The analysis of soil bacterial community composition showed that overall, 70% of bacterial community comprised *Proteobacteria*, *Bacteroidetes*, *Actinobacteria*, *Chloroflexi*, *Firmicutes*, *Acidobacteria,* and *Gemmatimonadetes*. About 8% of soil bacterial phylotypes were categorized as ‘unidentified’ (Figure 4A). Lower relative abundance of *Proteobacteria*, *Acidobacteria*, and *Gemmatimonadetes* was observed in response to MB application (S-UI). Abundances of *Proteobacteria* and *Acidobacteria* decreased from 36.1 ± 1.08 to 26.9 ± 0.93% and 3.5 ± 0.27 to 1.6 ± 0.35%, respectively, in treatment S-UI compared to the control. In treatment S-I_BC (augmented with biochar immobilized MB3R), abundances of these phylotypes were restored to 34 ± 1.26 and 3 ± 0.31%, respectively. Relative abundances of phyla *Bacteroidetes*, *Actinobacteria,* and *Firmicutes* were higher in the soil spiked with MB (S-UI). Bacterial phylotypes belonging to these phyla were 11.5 ± 1.03, 11.6 ± 0.71, and 0.69 ± 0.13% in control (un-spiked) soil, respectively, as compared to 22.0 ± 1.31, 14.7 ± 1.09 and 1.9 ± 0.28% in MB-contaminated soil, i.e., treatment S-UI. The relative abundance of *Bacteroidetes*, *Actinobacteria,* and *Firmicutes* was 17.7 ± 1.07, 13.1 ± 1.16, and 4.6 ± 0.61% in soil augmented with biochar immobilized bacterial consortium MB3R (S-I_BC).

**Figure 4:** **(A–C)** Overview of the relative populations of soil bacterial communities with respect to **(A)** phylum, **(B)** class, and **(C)** family under various treatments.

Among the phylum *Proteobacteria, Alphaproteobacteria*, *Betaproteobacteria,* and *Gammaproteobacteria* were the dominant classes with 20.7 ± 1.14,1.9 ± 0.38, and 14.0 ± 1.0% relative abundance in the control treatment, respectively (Figure 4B). MB contamination of soil (S-UI) reduced the abundances of *Alphaproteobacteria*, *Betaproteobacteria,* and *Gammaproteobacteria* to 14.7 ± 0.73, 1.0 ± 0.4, and 8.2 ± 0.62%, respectively. The relative abundance of these classes became higher (compared with the control) when MB-contaminated soil was augmented with MB3R immobilized on biochar (S-I_BC). Dominant classes of phylum *Acidobacteria* were *Acidobacteria_*Gp4 and *Acidobacteria_*Gp6. The populations of these classes decreased from 1.76 ± 0.33 to 0.71 ± 0.17% and 1.44 ± 0.31 to 0.69 ± 0.5% after MB addition in contrast to control. However, the relative abundance of *Acidobacteria_*Gp4 and *Acidobacteria_*Gp6 became higher (1.31 ± 0.26 and 1.59 ± 0.33% respectively) in treatment S-I_BC. Among the phylum *Bacteroidetes*, there was a significantly higher abundance of the class *Flavobacteria* in response to MB addition, while lower abundances of classes *Cytophagia* and *Sphingobacteria* were recorded in soil contaminated with MB. The abundance of bacteria belonging to both classes was rehabilitated in soil treated with MB3R and biochar.

In all treatments, the majority of *Proteobacteria* were related to the families *Sphingomonadaceae*, *Hyphomicrobiaceae*, and *Phyllobacteriaceae* (Figure 4C). Their abundances in control treatments were 7.7 ± 0.59, 1.96 ± 0.29, and 1.62 ± 0.35%, respectively, and were reduced to 1.76 ± 0.22, 0.92 ± 0.16, and 0.88 ± 0.12% in MB spiked uninoculated soil (S-UI). In soil augmented with MB3R immobilized on biochar, the relative abundance of *Sphingomonadaceae, Hyphomicrobiaceae,* and *Phyllobacteriaceae* increased to 6.47 ± 0.74, 1.62 ± 0.31, and 1.41 ± 0.21%, respectively.

## Discussion

The study aimed to assess the efficiency of native and biochar-immobilized bacterial consortium MB3R for remediation of MB-contaminated soil as well as restoration of bacterial community composition after an MB challenge. The *in-situ* MB-degrading capability of MB3R was enhanced significantly when immobilized onto biochar. This may be because of the high porosity and surface area of biochar which provide immobilized bacteria a safe environment within its pores, and increase their survival and activity by enhancing nutrient availability and inactivation of substances that can hinder microbial growth (Pietikainen et al., 2000; Steinbeiss et al., 2009). Furthermore, biochar can assist the transport of electrons among microorganisms and pollutants by activating persistent free radicals (Yu et al., 2015). Reduction in the toxicity of hazardous compounds due to the presence of biochar has already been suggested as a possible reason for enhanced proliferation of microbes and hence biodegradation of contaminants (Choppala et al., 2012). The present results are consistent with a previous study where enhanced degradation of cypermethrin (CP) was observed by immobilizing a CP-degrading bacterial consortium onto biochar (Liu et al., 2017). In another study, immobilization of *Corynebacterium variabile* HRJ4 on biochar improved the degradation of total petroleum hydrocarbons (Zhang et al., 2016). Other researchers reported the enhanced degradation of pollutants like polycyclic aromatic hydrocarbons (PAH) by inoculating the soil with bacteria immobilized onto biochar (Chen B. et al., 2012; García-Delgado et al., 2015).

The mathematical model used to determine MB degradation kinetics showed that MB degradation fits first-order equation. Previously, a number of researchers reported that microbial degradation of compounds like CP, beta-cypermethrin, and dimethyl phthalate followed first-order kinetics (Chen S. et al., 2012; Zhou et al., 2014; Akbar et al., 2015). In the present study, addition of the MB3R-biochar to soil resulted in the highest removal rate constant and shortest half-life of MB during amongst all other treatments (Table 3). Sites provided by the biochar for adsorption and oxidation/reduction reactions due to the presence of graphite structure can be the possible reason for the reduction of half-life and accelerated removal rate (Oh et al., 2013). In a previous study, the half-life of cypermethrin decreased significantly in the presence of biochar immobilized cypermethrin-degrading bacteria (Liu et al., 2017).

Three metabolites produced during biodegradation of MB by the consortium MB3R in minimal salt medium have been reported by our group (Wahla et al., 2019). The DA and DK are formed as a result of deamination and desulfuration of MB, respectively (Henriksen et al., 2002; Khoury et al., 2006). Further removal of the -NH_2_ group (deamination) from DK or removal of the -SCH_3_ group (desulfuration) of DA results in the formation of DADK (Mutua et al., 2016). In the present study, no MB metabolites were detected in the uninoculated treatments, i.e., S-UI and S-UI_BC, which might be due to a minimal degradation of MB. The detection of all three metabolites in inoculated treatments S-I and S-I_BC at all samplings depicted the involvement of MB3R in the transformation of MB. The decrease in concentrations of metabolites at 60 and 90 DAI as compared to 30 DAI provides evidence for further degradation of the aforementioned metabolites by MB3R in soil.

The analysis of 16S rRNA amplicon sequences of soil microbial communities indicated that application of MB significantly (*p* < 0.05) changed the microbial community structure but have minor effect on the overall microbial diversity. In response to MB, the relative abundance of some phyla like *Actinobacteria*, *Bacteroidetes,* and *Firmicutes* increased. Members of these phyla might be tolerant to MB and proliferate in the presence of MB due to reduced competition for space and available nutrients (Johnsen et al., 2001; Russell et al., 2011). In contrast, the relative abundance of *Proteobacteria*, *Acidobacteria,* and *Gemmatimonadetes* decreased in MB-spiked uninoculated soil (S-UI) as compared to the control. This change in the abundance of bacteria belonging to these phyla following exposure to MB may be due to the toxic effects of this pesticide. Pesticides can also cause an indirect suppression of the proliferation of some microbes by changing physio-chemical properties of their habitats (Johnsen et al., 2001; Schäfer et al., 2012). The decrease in the abundance of *Proteobacteria* in response to sulphonamides and sulfamethazine has been reported previously (Islas-Espinoza et al., 2012; Bai et al., 2019) which was in agreement with the results of the current study.

In the current study, we observed positive effects of the biochar-immobilized bacterial consortium MB3R on the abundance of bacterial communities, i.e., *Proteobacteria*, *Acidobacteria,* and *Firmicutes*. Apparently, under treatment P-I_BC, the soil microbial community structure was restored as it was similar to the control un-spiked soil. This might be due to the reduced toxicity, as almost 78% of the applied MB was degraded in this treatment. Also, biochar is reported for varying effects on soil prokaryotic communities. Some researchers have reported positive effects of biochar on the abundance of *Proteobacteria*, *Bacteroidetes*, *Actinobacteria*, *Gemmatimonadetes*, and *Planctomycetes* (Hu et al., 2014; Cheng et al., 2017; Meng et al., 2019), while in other studies, the abundance of *Proteobacteria*, *Acidobacteria*, *Firmicutes,* and *Bacteroidetes* was reduced in response to biochar application (Kolton et al., 2011; Ding et al., 2013; Wu et al., 2016).

### Practical implications of this study

The practical implications of the study would be effective application of the biochar immobilized MB-degrading bacterial consortium MB3R for remediation of MB in soil at point source contamination. It will be possible to get rid of contaminating MB residues and hence improve soil quality without any environmental risks. The process will also prove to be beneficial to farmers interested in organic farming as it will make it possible to get rid of the pesticide residues in their lands and hence the products. In future, study will be planned in microplots and fields at multiple locations to further assess if the process could be up-scaled for field application. Further, potential degradation genes of all the four bacterial strains will be identified by analyzing their whole genome sequences using the next generation sequencing approach. New biocarrier materials will also be identified for effective immobilization of MB-degrading bacterial strains for enhanced remediation of MB-contaminated sites.

## Conclusion

Microbial degradation of pesticides by bacteria has been widely reported and degrading strains have been identified, but their application for remediation of soil has been limited to only few reports, which is often due to low efficiency of bacteria in open environment and also availability of adequate carrier materials. Biochar was used as an easily available and environmentally friendly carrier material to immobilize the consortium MB3R, which not only enhanced the remediation efficiency but also helped to restore the microbial communities affected due to the MB-induced stress. In microcosms treated with MB3R immobilized on biochar, concentrations of metabolites produced during degradation of MB diminished toward the end of experiments, which indicates that further degradation of these metabolites to chemically simpler products took place. Augmentation with the consortium MB3R immobilized on biochar seems to be a promising approach for remediation of soils contaminated with metribuzin and to rehabilitate bacterial populations. Our results suggest that biochar can be used as effective carrier material for metribuzin-degrading bacteria. The application of this combination to agricultural soils may alter the fate and reduce the half-life of metribuzin by accelerating its degradation. Thus, MB3R immobilized biochar would be an effective approach for bioremediation of MB contaminated at point source contamination.

## Data availability statement

The data presented in the study are deposited in the GenBank repository, accession numbers are MG966499, MG966500, MG966501, and MG966502.

## Author contributions

AW, SI and ShA: supervision, resources, funding acquisition, formal analysis, investigation, writing-original draft, writing-review and editing. SaA and LA: statistical analyses, writing-original draft, writing-review and editing. ShA, SI and WI: project administration, data curation, methodology, software, writing-original draft, writing-review and editing. MF: methodology, formal analysis, writing-original draft, writing-review and editing. HA, AB, AA, SI: writing-original draft, writing-review and editing, funding acquisition, software. All authors contributed to the article and approved the submitted version.

## Funding

This work was funded by Institutional Fund Projects under grant no. (IFPIP: 702-130-1443), Ministry of Education in Saudi Arabia.

## Conflict of interest

The authors declare that the research was conducted in the absence of any commercial or financial relationships that could be construed as a potential conﬂict of interest.

## Publisher’s note

All claims expressed in this article are solely those of the authors and do not necessarily represent those of their affiliated organizations, or those of the publisher, the editors and the reviewers. Any product that may be evaluated in this article, or claim that may be made by its manufacturer, is not guaranteed or endorsed by the publisher.

## Footnotes

^1^ https://kasperskytte.shinyapps.io/shinyampvis/
